# Cost-Effectiveness of Interventions to Prevent Disability in Leprosy: A Systematic Review

**DOI:** 10.1371/journal.pone.0004548

**Published:** 2009-02-20

**Authors:** Natasja H. J. van Veen, Paul McNamee, Jan Hendrik Richardus, W. Cairns S. Smith

**Affiliations:** 1 Department of Public Health, Erasmus MC, University Medical Center Rotterdam, Rotterdam, Netherlands; 2 Health Economics Research Unit, Institute of Applied Health Sciences, University of Aberdeen, Aberdeen, United Kingdom; 3 Section of Population Health, School of Medicine & Dentistry, University of Aberdeen, Aberdeen, United Kingdom; Charité-Universitätsmedizin Berlin, Germany

## Abstract

**Background:**

Prevention of disability (POD) is one of the key objectives of leprosy programmes. Recently, coverage and access have been identified as the priority issues in POD. Assessing the cost-effectiveness of POD interventions is highly relevant to understanding the barriers and opportunities to achieving universal coverage and access with limited resources. The purpose of this study was to systematically review the quality of existing cost-effectiveness evidence and discuss implications for future research and strategies to prevent disability in leprosy and other disabling conditions.

**Methodology/Principal Findings:**

We searched electronic databases (NHS EED, MEDLINE, EMBASE, and LILACS) and databases of ongoing trials (www.controlled-trials.com/mrct/, www.who.int/trialsearch). We checked reference lists and contacted experts for further relevant studies. We included studies that reported both cost and effectiveness outcomes of two or more alternative interventions to prevent disability in leprosy. We assessed the quality of the identified studies using a standard checklist for critical appraisal of economic evaluations of health care programmes. We found 66 citations to potentially relevant studies and three met our criteria. Two were randomised controlled trials (footwear, management of neuritis) and one was a generic model-based study (cost per DALY). Generally, the studies were small in size, reported inadequately all relevant costs, uncertainties in estimates, and issues of concern and were based on limited data sources. No cost-effectiveness data on self-care, which is a key strategy in POD, was found.

**Conclusion/Significance:**

Evidence for cost-effectiveness of POD interventions for leprosy is scarce. High quality research is needed to identify POD interventions that offer value for money where resources are very scarce, and to develop strategies aimed at available, affordable and sustainable quality POD services for leprosy. The findings are relevant for other chronically disabling conditions, such as lymphatic filariasis, Buruli ulcer and diabetes in developing countries.

## Introduction

Leprosy is a leading cause of permanent disability among communicable diseases. An estimated three million people live with disability due to leprosy [1] and it is expected that up to one million people will continue to suffer from disability in the next decades [2]. The International Classification of Functioning, Disability and Health (ICF) defines disability as ‘an umbrella term for impairments, activity limitations and participation restrictions’ [3]. This definition goes beyond the concept of considering disability in medical terms only, and recognises the social context of disability. More than most other diseases, leprosy has a very negative image. People with visible disability fear stigmatization and discrimination, and experience serious psychosocial and economic problems [4]–[6].

One of the main components of leprosy programmes and research has been prevention of disability (POD). Interventions include: early detection and treatment of reactions and nerve damage, self-care interventions, health education, footwear programmes, and reconstructive surgery. More recently, the need for clear and sound guidance for leprosy control activities resulted in the organization of a technical forum by the International Leprosy Association (ILA). Their report, published in 2002, reviewed the existing literature for the effectiveness of important issues related to leprosy control, but did not address cost-effectiveness [7]. In 2006, a Consensus Development Conference on prevention of disability in chronically disabling conditions, such as leprosy, lymphatic filariasis, Buruli ulcer and diabetes was held. The main research theme of the conference was how to achieve universal coverage of essential POD interventions. One of the conclusions was that priority should be given to research that addresses issues of coverage and access [8].

In developing or low-income countries, cost-effective interventions often do not reach many of those who need them most. Achieving universal coverage usually means ‘going to scale’, defined as ‘a policy that builds on one or more interventions with known effectiveness and combines them into a programme delivery strategy designed to reach high, sustained, and equitable coverage, at adequate levels of quality, in all who need the interventions’. It assumes that the chosen interventions for scaling up are known to be feasible, affordable, and effective for implementation in the specific setting [9].

Evidence for the effectiveness of POD interventions in leprosy is limited. Recently, two systematic reviews have been published. One review assessed the effects of corticosteroids for treating nerve damage in leprosy [10] but did not find evidence from randomised controlled trials for a significant long-term effect of steroid therapy in improving either mild sensory nerve function impairment [11] or longstanding nerve function impairment [12].

The second review assessing the effects of interventions for skin damage in leprosy [13] found weak evidence favouring topical ketanserin over clioquinol cream or zinc paste [14] and topical phenytoin over saline dressing [15], [16] in ulcer healing. No evidence from randomised controlled trials for the effectiveness of self-care or educational interventions was found.

Cost-effectiveness data are even more limited, though the importance of cost-effectiveness analysis has been recognised. The ILA technical forum included a research question about which methods are most cost-effective, but did not answer this question in their report [7]. The consensus statement on POD mentioned that it would be more cost-effective to combine POD strategies and interventions for several related chronically disabling conditions in leprosy-endemic countries, and recommended further research on cost-effective methods to promote self-care and the use of appropriate footwear [8].

We assessed the existing literature on cost-effectiveness of POD interventions in leprosy as it was not clear which interventions were most cost-effective, using a standard checklist for economic evaluations and discussed the findings in the light of availability, affordability, and sustainability of POD interventions for leprosy and other chronically disabling conditions in developing countries.

## Methods

### Searching

In November 2008, a systematic search was done. We searched the NHS EED database (from 1994) using the search term: leprosy. We searched MEDLINE (from 1966), EMBASE (from 1980), and LILACS (from 1982), using the strategy in table 1. We searched databases of ongoing trials (www.controlled-trials.com/mrct/, www.who.int/trialsearch), we checked reference lists for any additional relevant studies, and we contacted experts in leprosy for ongoing studies or unpublished data. There were no language restrictions when we searched for publications.

**Table 1:** Search strategy for identifying economic evaluations of interventions to prevent disability in leprosy.

#	Term	Field
1	economics	MeSH Subheading
2	economic evaluation	title or abstract
3	cost-benefit analysis	title or abstract
4	cost-effectiveness analysis	title or abstract
5	cost-effective	title or abstract
6	cost-utility analysis	title or abstract
7	cost	title or abstract
8	costs	title or abstract
9	or/1–8	
10	leprosy	title or abstract
11	hansen's disease	title or abstract
12	hansen disease	title or abstract
13	or/10–12	
14	disability	title or abstract
15	disabled	title or abstract
16	deformity	title or abstract
17	deformed	title or abstract
18	impairment	title or abstract
19	impaired	title or abstract
20	neuritis	title or abstract
21	nerve damage	title or abstract
22	nerve function impairment	title or abstract
23	reaction	title or abstract
24	reactions	title or abstract
25	ulcer	title or abstract
26	eye damage	title or abstract
27	visual impairment	title or abstract
28	blindness	title or abstract
29	footwear	title or abstract
30	self-care	title or abstract
31	surgery	title or abstract
32	or/14–31	
33	9 and 13 and 32	

### Selection

We included studies that met the following criteria:

- assessing interventions to prevent disability in leprosy and
- comparing two or more competing alternatives and
- reporting both cost and effectiveness of the interventions compared

There were no restrictions on the type of study design when we searched for publications.

### Validity assessment

We assessed the quality of the studies, using a check-list from Drummond al. [17], consisting of ten essential questions, for critically appraising studies of economic evaluation of health care programmes (see table 2). With respect to question 10 (did the presentation and discussion of study results include all issues of concern to users), we focussed on availability, affordability, and sustainability. Availability includes issues of coverage and access, affordability means that each of the parties involved is able and willing to pay for a given health care programme or intervention, and sustainability refers to long-term strategies for sustaining health care programmes.

**Table 2:** Check-list for assessing economic evaluations.

1	Was a well-defined question posed in answerable form?
2	Was a comprehensive description of the competing alternatives given?
3	Was the effectiveness of the programmes or services established?
4	Were all the important and relevant costs and consequences for each alternative identified?
5	Were costs and consequences measured accurately in appropriate physical units?
6	Were costs and consequences valued credibly?
7	Were costs and consequences adjusted for differential timing?
8	Was an incremental analysis of costs and consequences of alternatives performed?
9	Was allowance made for uncertainty in the estimates of costs and consequences?
10	Did the presentation and discussion of study results include all issues of concern to users?

From: Drummond al. 2005 (17).

### Data abstraction and study characteristics

One author (NvV) extracted the relevant data (e.g. type of study design, interventions, outcome measures) from the eligible studies and a second author (PMN) checked the data. The authors discussed discrepancies between themselves. Missing data were obtained from study authors where possible. The authors were not blinded to the names of study authors, journal or institutions.

### Quantitative data synthesis

For studies with a similar type of POD intervention, we planned to calculate standardised estimates of the cost per disability-adjusted life-year (DALY). Where it was not possible to pool data, we summarised the cost-effectiveness data for each study.

## Results

### Flowchart

The electronic searches found 62 citations to potentially relevant studies. Two further potentially eligible studies were found from reference lists of included studies and reviews. Correspondence with experts in leprosy and searching of grey literature revealed another two potentially relevant studies. We identified seven possible studies of economic evaluation. The search of the ongoing trial registers did not reveal any ongoing trials. We excluded four studies. One study was a review paper describing only costs of different components of a global leprosy elimination programme [18]. The second study modelled the productivity gains if deformity would be eliminated [19]. The third study assessed only the cost of offering disability care either through community volunteers or leprosy workers at the clinic [20]. The fourth study was an unpublished report describing guidelines for doing a systematic cost analysis in leprosy control programmes [21]. Figure 1 shows the selection process of the studies.

**Figure 1:** Flowchart of selection process.

### Study characteristics

We included three studies. Two studies were small, single-centre randomised controlled trials. One trial (Seboka 1996) assessed the cost-effectiveness of canvas shoes compared to plastazote shoes in terms of cost per ulcer healed or prevented [22]. The other trial (Ravi 2004) compared the cost of ambulatory care to hospitalisation in the management of neuritis and used the number of days needed to return to work as primary outcome of effectiveness [23]. The third study (Remme 2006) reviewed the effectiveness of interventions and calculated cost of existing interventions per DALY averted [24]. It was published in the second edition of the World Bank publication ‘Disease Control Priorities in Developing Countries’ [25]. Table 3 summarises the general characteristics of the three studies.

**Table 3:** General characteristics of included studies.

Study ID	Seboka 1996	Ravi 2004	Remme 2006
Design	Randomised controlled trial	Randomised controlled trial	Model-based study
Randomisation procedure	Randomisation by day of attendance to clinic	Randomisation by computerized random numbers table	Not applicable
Setting	Foot-care clinic near Sheshemane, Ethiopia	Skin and leprosy department of tertiary level hospital in Tamilnadu, India	Not applicable
Time of study	November 1994 to November 1995	October 1999 to March 2001	Not applicable
Number of patients	70	26	Not applicable
Inclusion	Leprosy patients with deformed and anaesthetic feet	Leprosy patients with neuritis <6 month duration due to type 1 or type 2 reaction	Not applicable
Male/female	28/40 (2 unknown)	23/3	Not applicable
Mean age (range)	Not described (unclear)	31 (15–49) (exp)^1^; 41 (19–60) (cont)^2^	Not applicable
Lost to follow-up	2 (cont)^2^	4 (2 exp, 2 cont)^1^ ^2^	Not applicable
Interventions	Experimental group (n = 40): canvas shoes	Experimental group (n = 13): ambulatory care: education and steroid therapy (mean duration 4.3 months)	Treatment for reactions and ulcers, footwear and self-care education, reconstructive surgery
	Control group (n = 30): plastazote shoes	Control group (n = 13): hospitalisation for 2 weeks plus steroid therapy (mean duration 4.5 months)	Comparing total cost and benefits of existing interventions, starting from zero
Outcomes	Healing of existing ulcers	Number of days needed to return to work after stipulated period of admission or rest (2 weeks)	Cost per DALY averted
	Prevention of ulceration	Mean cost per patient	Average cost of POD per new leprosy case with disability
	Acceptability of shoes	Improvement in quality of life score	
	Durability of shoes	Improvement in sensory and motor score	
	Cost-effectiveness of shoes		
Timing of outcome assessment	One year after start from study	At the end of steroid therapy	Not applicable

1 exp: experimental group.

2 cont: control group.

### Validity assessment

For a critical appraisal of the studies, we answered all ten questions of the standard checklist [17] for each of the studies identified. The results of the critical assessment are summarised in table 4.

**Table 4:** Quality of included studies.

	Study ID		
**Criteria**	**Seboka 1996**	**Ravi 2004**	**Remme 2006**
1) Well-defined question stated?	no^a^	no^a^	no^a^
2) Description of alternatives given?	yes	yes	yes
3) Evidence of effectiveness established?	yes	yes	yes
4) Relevant costs and outcomes identified?	no^b^	not sure^c^	no^d^
5a) Costs measured accurately?	no^e^	yes	no^f^
5b) Outcomes measured accurately?	no	yes	yes
6a) Costs valued credibly?	yes	yes	yes
6b) Outcomes valued credibly?	not applicable^g^	not applicable^g^	not sure^h^
7a) Costs discounted?	not applicable^i^	not sure^j^	yes
7b) Outcomes discounted?	not applicable^i^	not sure^j^	yes
8) Incremental analysis performed?	no	no	no
9) Sensitivity analysis performed?	no	no	no
10a) Issue of availability addressed?	no	no	no
10b) Issue of affordability addressed?	no	no	no
10c) Issue of sustainability addressed?	yes	no	no

a no viewpoint for the analysis stated.

b only cost of shoes included.

c not sure whether shared costs were taken into account.

d only direct health care cost included.

e wholesale price or estimated cost of pair of shoes.

f estimated costs based on limited published data and expert opinion.

g outcomes in natural units.

h disability weights of DALY based on consensus of experts, but not on patient's values or preferences.

i all costs and consequences occurred within one year.

j not sure whether discounting was done.

#### 1. Was a well-defined question posed in answerable form?

The three studies did not state explicitly the viewpoint for the analysis (e.g. a specific provider or providing institution, the patient or groups of patients, a third-party payer, or society). Seboka 1996 implicitly referred to third-party payers (donors) with respect to long-term costs. Ravi 2004 estimated costs incurred by the health sector and the patient, and indirect costs due to lost working days, implying a societal perspective for the analysis. Remme 2006 included only direct costs to the health system of delivering interventions.

#### 2. Was a comprehensive description of the competing alternatives given?

Seboka 1996 compared two types of protective footwear, canvas shoes and plastazote or moulded shoes. Ravi 2004 assessed neuritis management through either ambulatory care or hospitalisation. Patients in the in-patient group were admitted for two weeks and were monitored in the ward for complications of steroid therapy. Patients receiving ambulatory care were educated regarding the complications of steroids and were advised rest at home for 2 weeks. Remme 2006 reviewed several existing POD interventions, compared to doing nothing.

#### 3. Was the effectiveness of the programmes or services established?

Evidence of effectiveness of footwear and neuritis management came from the trials itself (Seboka 1996 and Ravi 2004 respectively). Remme 2006 reviewed the literature for the effectiveness of POD interventions. Early case detection and treatment were considered as the most effective interventions to prevent disability in leprosy, and self-care as the main strategy to prevent worsening of impairments.

#### 4. Were all the important and relevant costs and consequences for each alternative identified?

Seboka 1996 included only the wholesale price for which the canvas shoes were purchased. Plastazote shoes were provided free-of-charge for the purpose of this study. The cost of organizing and operating the footwear service or the cost to the patient and family for follow-up visits was not measured. Ravi 2004 collected data on different cost categories, covering direct medical costs (e.g. examinations, medication, in-patient care), direct non-medical costs (e.g. transport and food of visitors and patients) and indirect costs (e.g. working days and wages lost), but it was unclear as to whether shared costs were taken into account. Remme 2006 estimated only the direct health care cost of delivering interventions.

Seboka 1996 used programme specific outcome measures of effectiveness (change in ulcer size, the acceptability, usefulness and durability of the footwear), but no generic quality of life outcome. The occurrence of adverse effects was not explicitly addressed, but the study did report that at least one out of five subjects in the plastazote group, who were initially ulcer-free, developed ulcers due to ill-fitting shoes. The primary outcome in Ravi 2004 was the number of days needed to return to work and this was considered a surrogate marker for effectiveness of treatment and well-being of the patient. Secondary outcomes were: mean cost per patient, improvement in nerve function scores and quality of life scores. None of the patients reported any significant adverse effects of steroid therapy. Remme 2006 used a generic outcome measure, the disability-adjusted life years (DALYs) and did not report on adverse effects.

#### 5. Were costs and consequences measured accurately in appropriate physical units?

The costs in Seboka 1996 were straightforward, but inaccurate; the wholesale price or estimated cost of a pair of shoes. Ravi 2004 calculated costs by multiplying the quantities of the resources used and the unit cost of each resource (e.g. cost of each examination, bed and nursing cost, transportation cost). Remme 2006 measured cost as cost of an intervention per patient. Costs were estimated from limited published cost data, programme expenditure data, and expert opinion.

Seboka 1996 measured the primary outcome in natural units; the number of ulcers healed or prevented. It was unclear what scale or score was used to measure acceptability and usefulness of the footwear. Ravi 2004 measured the primary outcome, the number of days needed to return to work, from the stipulated period of rest or admission. Improvement in nerve function was measured as a mean score using graded nylon filaments (score per nerve) and the Medical Research Council (MRC) scale (0–5 score per nerve). Quality of life was measured as a mean score using a questionnaire (20 questions, maximum score of 106) derived from the WHO QOL Global pool of questions. Remme 2006 measured the outcome in DALYs.

#### 6. Were costs and consequences valued credibly?

Seboka 1996 reported the prevailing wholesale price of a pair of canvas shoes in US dollars. Ravi 2004 reported costs in local currency (Indian rupees) based on prevailing prices. Remme 2006 converted cost estimates to US dollars 2000.

Seboka 1996 and Ravi 2004 measured the primary outcome in natural units, which does not require valuation of benefits in money terms. Remme 2006 valued outcomes in DALYs. The disability weights used to value the duration and severity of a particular disease or condition have been criticised, because these were established by expert opinion and consensus [26]. For leprosy, a disability weight of 0.152 was given to disabling leprosy and a weight of 0.000 to a leprosy case without disability [27]. These weights are likely to be underestimated, since they will not adequately capture all the disability resulting from leprosy, such as the major psychosocial impact of leprosy on the lives of leprosy patients, regardless of having disability or not [24].

#### 7. Were costs and consequences adjusted for differential timing?

Because Seboka 1996 was a one-year trial and all the costs and consequences occurred within a one-year period, no discounting was needed. The trial of Ravi 2004 had a duration of 1.5 years. The study did not report on discounting. In Remme 2006 discounting of costs was done using a 3% rate. The DALY incorporates a constant annual discount rate of 3% for outcomes [28].

#### 8. Was an incremental analysis of costs and consequences of alternatives performed?

Seboka 1996 and Ravi 2004 did not perform an incremental analysis. Although the canvas shoes and ambulatory care intervention had lower costs and higher effectiveness compared to the plastazote shoes and hospitalisation intervention respectively, no information on a statistically significant difference between the two competing alternatives was given. Remme 2006 calculated the average cost-effectiveness of existing interventions.

#### 9. Was allowance made for uncertainty in the estimates of costs and consequences?

None of the studies performed a sensitivity analysis.

#### 10. Did the presentation and discussion of study results include all issues of concern to users?

Availability: none of the studies discussed the issue of coverage and access.

Affordability: none of the studies discussed whether all parties involved would be able and willing to pay for POD programmes.

Sustainability: Seboka 1996 mentioned that the cost of providing footwear to patients for many years may be costly and will require long-term commitment from donors. The other studies did not discuss issues of sustainability.

### Quantitative data synthesis

We summarised the cost-effectiveness data for each study, because it was not possible to pool the data for calculating standardised estimates of the cost per disability-adjusted life-year (DALY). Seboka 1996 calculated the cost-effectiveness of canvas shoes compared to plastazote shoes to prevent and heal ulcers in leprosy patients with deformed and anaesthetic feet. The average cost per ulcer healed or prevented over a one-year period was $24.4 and $44.7 respectively. Additional information about the results of the plastazote group was obtained from one of the authors. The average cost per ulcer healed or prevented over a one-year period was at minimum $160 and $373 respectively.

Ravi 2004 calculated costs and effectiveness of ambulatory care compared to hospitalisation in the management of neuritis due to reactions in leprosy patients. The total mean cost per patient was approximately 7,234 rupees for ambulatory care versus 25,740 rupees for in-patient care. On average, patients receiving ambulatory care returned to work after 19.5 days, while hospitalized patients needed 66.8 days to return to work. Additionally, the study measured quality of life, but results for only 17 out of 26 patients were available. QOL scores improved in both groups, but the study did not find a significant mean difference in the pre- and post-treatment QOL scores between the two groups.

Remme 2006 estimated the average cost of POD for each new case of leprosy detected with disability at $44.10. The cost per DALY was calculated assuming a 25% self-cure rate, an average age of onset of 27, a disability weighting of 0.152, a life expectancy at age 25–29 of 44.75 (India data), and a 90% success rate. The cost per DALY for patients needing treatment for reactions and ulcers was estimated at $7, for those needing footwear and self-care education at $75, for those needing reconstructive surgery at $110.

## Discussion

### Summary of main findings

Evidence for cost-effectiveness of POD interventions for leprosy is scarce. We found three studies; two were small, single-centre randomised controlled trials and one was a model-based review study. One trial found that canvas shoes were more cost-effective than plastazote shoes in healing and preventing ulcers and the other trial showed that ambulatory care was more cost-effective (lower cost and earlier return to work) compared to hospitalisation in the management of neuritis. The model-based study estimated the cost of POD interventions per DALY averted between $7 and $110. None of the studies met all the quality criteria for economic evaluations. The cost perspective of the analysis, relevant and accurate costs, analysis of uncertainty in estimates, and issues of availability, affordability and sustainability were inadequately reported or addressed in the studies.

### Generalizability

Generalizability of the findings is limited. The two trials [22], [23] were conducted in a single centre and used prevailing or local prices to calculate costs. The economic evaluation was carried out alongside a randomised controlled trial and it has been argued that economic outcomes from such trials may differ significantly from usual practice or care [17]. The model-based study [24] stated that costs were likely to differ country by country and that the cost estimates should only be considered indicative, as they were based on limited published data and expert opinion. The cost of prevention of disability per new leprosy case with disability was expected to be higher than the estimate due to a backlog of old leprosy cases with disability, and this cost will be influenced by the numbers of multibacillary leprosy patients and the levels of disability in different settings and countries. The cost-effectiveness outcomes were also likely to vary, because these were based on limited effectiveness data, and the application of a disability weight of 0.152 to all patients may overestimate the benefits of interventions.

### Issues of concern

One of the criteria for critically assessing economic evaluations was whether studies discussed all issues of concern. We focussed on issues of availability, affordability and sustainability, since these are current challenges in resource-poor countries and for neglected tropical diseases. Few studies have addressed one of these issues. Whilst self-care appears to be an effective, affordable and sustainable intervention to prevent disability in leprosy or lymphatic filariasis, when initially taught and supervised by general health staff [29]–[31], we are not aware of evidence that has documented the cost-effectiveness of self-care strategies. The ILA technical forum report highlighted the need for sustainable leprosy services through integrated general health services and provided basic requirements for this process, such as involvement, commitment and collaboration of the different stakeholders and health staff, strengthening of health systems, and careful planning [7]. Also, patients should be adequately informed about the availability of existing POD services [32].

Achieving universal coverage would require cost-effective POD interventions that can be delivered at adequate quality levels to all who need them and for as long as needed. Strategies for going to scale need to consider the context or setting of implementation (e.g. skilled staff and resources available, burden of disease, benefits to others than target group), the balance between quality and coverage levels, the choice of the health delivery system (e.g. general health services, disease-specific programmes, community-based health workers, or mix of alternatives), costs involved (e.g. strengthening health systems), and longer-term planning [9].

### Strengths of the study

This is the first study that critically and systematically reviewed the existing literature on cost-effectiveness of interventions to prevent disability in leprosy. The search process was elaborate and to our knowledge no other studies were available for the review. We used a standard checklist to appraise the quality of economic evaluations of health care programmes and health interventions.

### Limitations of the study

It is possible that not all of the relevant studies have been included in this review, and that we failed to find some unpublished ones. We contacted several experts in leprosy, but this did not reveal any unpublished or ongoing studies. We were not able to compare the cost-effectiveness of similar interventions or calculate standardised outcome estimates, due to lack of data on costs and effectiveness outcomes. Recently, two questionnaires on aspects of quality of life were developed and validated for chronically disabling conditions, such as leprosy, polio, spinal cord injuries and diabetes. One questionnaire (SALSA) measures limitations in daily activities [33], and the other one (Participation Scale) assesses perceived restrictions in social participation [34]. These questionnaires may be useful in assessing and comparing the effects of interventions and programmes for chronic and disabling conditions on patient-perceived changes in quality of life.

In conclusion, cost-effectiveness analysis should play an important role in the informed debate about issues of availability, affordability and sustainability of health care programmes or health interventions for chronically disabling diseases, such as leprosy, lymphatic filariasis, Buruli ulcer and diabetes, in resource-poor countries. It is recommended that future economic evaluation studies better define the cost perspective, the relevant alternatives, costs and outcomes of POD interventions, including adverse effects, and potentially uncertain variables, and to address issues of availability, affordability and sustainability. Future studies are needed to establish the cost-effectiveness of POD interventions and these should adhere to standard guidelines for economic evaluations.
